# Exosomal lncRNA HNF1A-AS1 affects cisplatin resistance in cervical cancer cells through regulating microRNA-34b/TUFT1 axis

This article has been retracted.

**DOI:** 10.1186/s12935-019-1042-4

**Published:** 2019-12-03

**Authors:** Xiaoqiong Luo, Jingxi Wei, Feng-lian Yang, Xiao-xia Pang, Feng Shi, Yu-xia Wei, Bi-yun Liao, Jun-li Wang

**Affiliations:** 1 Center of Reproductive Medicine, Affiliated Hospital of Youjiang Medical College for Nationalities, Zhongshan Second Road 18th, Baise, 533000 Guangxi China; 2 Youjiang Medical College for Nationalities, Baise, 533000 People’s Republic of China

**Keywords:** Cervical cancer, Exosomes, LncRNA HNF1A-AS1, microRNA-34b, TUFT1, ceRNA

## Abstract

**Background:**

There is growing evidence of the role of long non-coding RNAs (lncRNAs) in cervical cancer (CC). The objective was to discuss whether exosomal lncRNA HNF1A-AS1 impacted drug resistance in CC via binding to microRNA-34b (miR-34b) and regulating TUFT1 expression.

**Methods:**

The expression of HNF1A-AS1 in normal cervical epithelial cells, cisplatin (DDP)-sensitive cell line (HeLa/S) and DDP-resistant cell line (HeLa/DDP) cells were detected. HeLa/S and HeLa/DDP cells were interfered with HNF1A-AS1 to determine IC_50_, proliferation, colony formation and apoptosis of CC cells. The exosomes were isolated and identified. Subcellular localization of HNF1A-AS1, expression of miR-34b and TUFT1 in receptor cells were also verified. The binding site between HNF1A-AS1 and miR-34b, together with miR-34b and TUFT1 were confirmed. Tumorigenic ability of cells in nude mice was also detected.

**Results:**

HNF1A-AS1 was upregulated in DDP-resistant cell line HeLa/DDP. Silencing HNF1A-AS1 suppressed CC cell proliferation and promoted its apoptosis. HNF1A-AS1 was found to act as a competing endogenous RNA (ceRNA) of miR-34b to promote the expression of TUFT1. Exosomes shuttled HNF1A-AS1 promoted the proliferation and drug resistance of CC cells and inhibited their apoptosis by upregulating the expression of TUFT1 and downregulating miR-34b. Furthermore, suppressed exosomal HNF1A-AS1 in combination with DDP inhibited tumor growth in nude mice.

**Conclusion:**

Our study provides evidence that CC-secreted exosomes carrying HNF1A-AS1 as a ceRNA of miR-34b to promote the expression of TUFT1, thereby promoting the DDP resistance in CC cells.

## Background

Cervical cancer (CC) is the fourth common cancer among women, accounting for almost 7.5% of female cancer deaths in the world [1]. CC is still the most common cancer in Eastern and Middle Africa [2]. It is reported that human papillomavirus (HPV) is one of the main causes of CC [3], and other exogenous risk factors that have sexual relations with several partners, or early sexual behavior, as well as smoking, could also contribute to CC risk [4]. There is a possible impact of genetic factors to the risk of HPV infection progression to cervical precancer and CC [5]. It has been suggested that the standard primary treatment of CC includes radiotherapy (RT), or radical hysterectomy with pelvic lymph node dissection (RHND), or a combination of RT and platinum-based chemotherapy [6]. Cisplatin (DDP) is a widely-used potent chemotherapeutic drug for the treatment of CC, while its effectiveness is restricted by the resistance development [6]. Consequently, the recognition of novel prognostic markers might be helpful for offering more personalized medical treatment for CC.

Long non-coding RNAs (lncRNAs) is a kind of non-coding transcript with more than 200 nucleotides, which lacks the potential of protein coding [7]. Exosomes has great effects on the cell signal transmission and communication which is formed in the endosome [8]. LncRNAs were found in the exons and further demonstrated their true biological function in tumor development and drug resistance [9]. Long non-coding RNA HNF1A antisense RNA 1 (lncRNA HNF1A-AS1) is a natural antisense transcript of HNF1A, which is on chromosome 12q24.31 and has a total length of 2455 nucleotides [10]. Abnormal expression of HNF1A-AS1 has been reported in sundry human cancers and HNF1A-AS1 could as a tumor inducer gene or tumor suppressor gene [11]. A study has reported that restoration of HNF1A-AS1 accelerated cell proliferation, invasion, cell cycle and migration of non-small cell lung cancer cells in vitro [12]. Another study revealed that overexpression of HNF1A-AS1 forecasted poor prognosis for oral squamous cell carcinoma patients [13]. LncRNAs has been confirmed as competition for microRNA (miRNA) sponges in competing endogenous RNA (ceRNA) networks, which is participate in modulates the expression of miRNA [14]. miRNA is an endogenous small non-coding RNA molecule (19–22 bases in length), which binds to the incomplete sequence homology site of mRNA’s 3′-untranslated region (3′-UTR), and leads to the degradation or inhibition of protein translation [15]. There is a study highlighting the role of miR-34b in regulating the proliferation and apoptosis of CC cells [16]. Tuftelin1 (TUFT1) is an acidic protein that exists in the developmental and mineralization tissues of teeth [17]. It is reported in a study that in breast cancer tissues, the expression of TUFT1 increased significantly [18]. A study has demonstrated that TUFT1 is a factor in the poor prognosis of various cancers [19]. Based on the aforementioned evidence, our study was performed to discuss whether CC-derived exosomes carrying HNF1A-AS1 could act as a competing endogenous RNA (ceRNA) of miR-34b to increase the expression of TUFT1, thereby affecting DDP resistance, proliferation and apoptosis in CC cells. Thus, a series of experiments were performed in this study to justify the hypothesis.

## Materials and methods

### Ethics statement

The study was approved by the Ethics Committee of Center of Reproductive medicine, Affiliated hospital of Youjiang Medical College for Nationalities (Ethical number: 201801002). All animal experiments were in compliance with the recommendations in the Guide for the Care and Use of Laboratory Animals of the National Institutes of Health.

### Cell culture

Human normal cervical epithelial cells HcerEpic, DDP-sensitive CC cell line HeLa/S and DDP-resistant cell line HeLa/DDP were bought from the Cell Bank of the Chinese Academy of Sciences (Shanghai, China). And then, they were cultured by Roswell Park Memorial Institute (RPMI) 1640 medium with 10% fetal bovine serum (FBS) and penicillin-streptomycin (Gibco by Life technologies, Grand Island, New York, USA), and placed in an incubator of 37 °C, 5% CO_2_. Cell detachment was performed with 0.25% trypsin and passaged in an amount of 1:3. Cells were seeded in a 6-well plate, and when the confluence reached 70% to 80%, cells in the logarithmic growth phase were used in subsequent experiments.

### Exosomes separation and identification

The transfected CC cells were inoculated into RPMI 1640 medium containing 10% FBS without exosomes, and cultured in a 37 °C, 5% CO_2_ incubator. Cell supernatants were collected 3 days later and centrifuged to remove cell debris. The exosomes were extracted according to the instructions of Hieff™ Quick exosome isolation kit (41201ES50, YEASEN, Shanghai, China). The supernatant and exosome separation reagent were added into the Eppendorf (EP) tube with a proportion of 2:1 overnight, and then centrifuged at 100,00*g*, 4 °C for 1–2 h. The supernatant was removed and the precipitate was the exosomes. According to the volume ratio of 10:1 for the starting culture and resuspension, phosphate buffered saline (PBS) (0.01 M, pH 7.4) was added for resuspension. Resuspended exosomes (30 μL) was placed in EP tubes, and an equal volume of radioimmunoprecipitation assay (RIPA) buffer was added, and then placed on ice. The exosomes was lysed for 10 s by microwave for 2 times. Lastly, the concentration of protein in the exosomes was measured by bicinchoninic acid (BCA) quantification kit (Beyotime Biotechnology, Nantong, China). Exosome markers CD63, CD9, and CD81 were verified by western blot analysis, and exosomal morphology was observed by a transmission electron microscope (TEM) (JEM-1010, JEOL, Tokyo, Japan). Dynamic light scattering was used to detect the diameter of the exosomes by using the Zetasizer Nano-ZS90 (Malvern Instrument, Worcestershire, UK), with an excitation wavelength of λ = 532 nm. Exosomes were diluted to a suitable optical signal detection level (1:50 ratio) with 0.15 M NaCl and mixed for detection. Finally, exosomes secreted by CC cells were obtained.

### Exosomes labeling and uptake of the exosomes

PKH67 fluorescent cell membrane labeling kit were available from Sigma-Aldrich (SF, CA, USA). Exosomes were naturally thawed on ice with a final volume of 100 μL. Exosomes suspension was mixed with 400 μL diluent C and named as exosomes mixture, while PHK67 (2 μL) was mixed with 500 μL diluent C and then named as PKH67 mixture. Exosomes mixture was mixed with PKH67 mixture and placed for 3 min. FBS (1 mL) was added into the mixture and placed for 1 min. The mixture was mixed with 2 mL RPMI 1640 medium and centrifuged at 100,000×*g* for 2 h. The supernatant was discarded. The mixture was suspended with proper amount of PBS and centrifuged at 100,000×*g* for 2 h and repeated for 3 times. The mixture was suspended and precipitated with 100 μL PBS to obtain the exosomes labeled by PKH67. Exosomes labeled by PKH67 was co-cultured with recipient cell HeLa/S and incubated for 24 h. Then HeLa/S cells were fastened, and sealed, and the nucleus was dyed with 4′,6-diamidino-2-phenylindole (DAPI). The expression of PKH67 in HeLa/S cells was observed by a laser confocal microscope.

### Cell grouping and transfection

In order to observe the role of HNF1A-AS1 in drug resistance of CC, we interfered with the expression of HNF1A-AS1 in DDP sensitive cell line HeLa/S and drug resistant cell line HeLa/DDP. HeLa/S and HeLa/DDP cells were distributed into two groups: small hairpin RNA (sh)-negative control (NC) group: cells transfected with sh-HNF1A-AS1 plasmid NC; sh-HNF1A-AS1 group: cells transfected with sh-HNF1A-AS1 plasmid. In order to further study whether the drug resistant exosomes promoted drug resistance through modulating expression of HNF1A-AS1, the effect of the exosomal HNF1A-AS1 on the sensitive cells was studied by establishing a co-culture model. HeLa/S cells were assigned into NC-exo group: HeLa/DDP transfected with overexpression (oe)-HNF1A-AS1 plasmid NC labeled by Cy3 was co-cultured with HeLa/S cells; HNF1A-AS1-exo group: HeLa/DDP transfected with oe-HNF1A-AS1 plasmid labeled by Cy3 was co-cultured with HeLa/S cells. HNF1A-AS1 plasmid and its NC, oe-HNF1A-AS1 plasmid labeled by Cy3 and its NC were available from Guangzhou RiboBio Co., Ltd. (Guangdong, China). HNF1A-AS1 plasmid and its NC, oe-HNF1A-AS1 plasmid labeled by Cy3 and its NC were transfected in strictly accordance with the instructions of Lipofectamine™RNAiMAX (Invitrogen, Carlsbad, CA, USA).

### Establishment of cell co-culture model

After 36 h transfection of elevated HNF1A-AS1, CC resistant cells were collected and inoculated with 1 × 10^5^ cells/well into the apical chamber of Transwell culture plate. The complete medium was supplemented to 300 μL. CC resistant cells were seeded into the apical chamber of Transwell 1 day in advance. The density of the cell plate was 1 × 10^5^ cells/well, and 3 parallel wells were set up in each group. After 24 h of co-culture in the apical and basolateral chambers, the entry of Cy3-HNF1A-AS1 into CC sensitive cells was observed under a FSX100 biocavitary navigator. At the same time, the CC sensitive cells were collected and the total RNA was extracted. Reverse transcription quantitative polymerase chain reaction (RT-qPCR) was utilized for detecting the HNF1A-AS1 expression.

### 3-(4, 5-dimethylthiazol-2-yl)-2, 5-diphenyltetrazolium bromide (MTT) assay

The cells were cultured in 96-well plates at the density of 1 × 10^4^ cells/well and cultured overnight at 37 °C and 5% CO_2_. The cells were treated with 0, 50, 100, 200, 400, 800 μg/mL DDP for 24 h in the medium with 10% FBS. IC_50_ of DDP was simultaneously detected. Then, cells were incubated with MTT solution (10 μL, 0.5 mg/mL) for 4 h. Dimethyl sulfoxide (DMSO) (200 μL) was added to terminate the reaction and incubated with cells at 37 °C for 15 min. The optical density (OD) value at 490 nm wavelength was observed by a microplate reader (Bio-Rad, Hercules, CA, USA).

### 5-ethynyl-2′-deoxyuridine (EdU) assay

The cells were cultured in a 96-well plate at 4 × 10^3^ cells/well, when reached 80% confluence, the cell proliferation was measured using an EdU detection kit (RiboBio, Guangzhou, China). After discarding the original medium, the cells were incubated with 100 μL 50 μm EdU medium (diluted with a cell culture medium at 1000:1) at 37 °C for 2 h, and washed twice with PBS (5 min per time). Cells were fixed with 50 μL 4% paraformaldehyde for 30 min and incubated with 50 μL 2 mg/mL glycocoll for 5 min. Cells were incubated with 100 μL 0.5% Triton X-100 penetrant for 10 min, washed with PBS (0.01 M, pH 7.4) for 5 min, and incubated in the dark with 100 μL 1× Apollo^®^ staining reaction for 30 min at room temperature, then infiltrated and decolorized with methanol. Lastly, the cells were stained with DAPI and examined by a Leica laser confocal microscope (Leica, Carl Zeiss, Jena, Germany).

### Colony formation assay

The transfected cells were seeded in a 6-well plate with 400 cells per well. Seven to fourteen days later, the culture was terminated after the colonies could be observed by the naked eye. Then the medium was absorbed and rinsed twice with PBS (0.01 M, pH 7.4). The cells were fixed by methanol for 30 min and stained with 0.1% crystal violet staining solution. Finally, colony imaging was counted to calculate the rate of cell colony formation.

### Flow cytometry

After 48 h of transfection, the cells were collected in the flow tube after detached with 0.25% trypsin (exclusive of ethylene diamine tetraacetic acid) (PYG0107, Boster, Wuhan, Hubei, China), and centrifuged at 1000 rpm for 10 min. Cold PBS (0.01 M, pH 7.4) was used to wash the cells 3 times, the supernatant was discarded by centrifugation. Annexin-V-fluorescein isothiocyanate (FITC), propidium iodide (PI), and 4-(2-hydroxyethyl)-1-piperazineëthanesulfonic acid (HEPES) buffer (0.01 M, pH 7.4, Beijing BioDee BioTech Co., Ltd., Beijing, China) were matched to AnnexinV FITC/PI staining solution at a ratio of 1:2:50 referring to the instructions of Annexin-V-FITC cell apoptosis detection kit (K201-100, BioVision, Palo Alto, USA). The 1 × 10^6^ cells were resuspended by 100 µL staining solution and incubated for 15 min, then mixed with 1 mL HEPES buffer. The fluorescence of FITC and PI was detected at the wavelength of 488 nm through a 515 or 620 nm bandpass filter, respectively, and the cell apoptosis was detected. The determination criteria of results: Annexin V was the transverse axis and the PI was the vertical axis; the upper left quadrant was (Annexin V-FITC)−/PI+, cells in this area were necrotic cells, while this area may included a small number of non-viable apoptotic cells, even mechanically damaged cells; the upper right quadrant was (AnnexinV-FITC)+/PI+, cells in this area were non-viable apoptotic cells; the lower right quadrant was (AnnexinV-FITC)+/PI−, cells in this area were viable apoptotic cells; the lower left quadrant was (AnnexinV-FITC)−/PI−, cells in this area were living cells. Apoptosis rate = [(viable apoptotic cells + non-viable apoptotic cells)/total number of cells] 100%.

### RNA-fluorescence in situ hybridization (FISH) assay

FISH technique was applied for verifying the subcellular localization of HNF1A-AS1 in cells. Following the instructions of Ribo™lncRNA FISH Probe Mix (Red) (RiboBio Co., Ltd., Guangzhou, China), the cover plate was placed in a 24-well plate and cells were inoculated with 6 × 10^4^ cells/well, so that the cells reached about 80% confluence. The glass was removed, and the cells were fixed with 4% paraformaldehyde (1 mL) at room temperature. Premixed solution (250 μL) was added after treated with protease K, glycine and acetylation reagent. Next, cells were incubated at 42 °C for 1 h. LncRNA HNF1A-AS1 (250 µL, 300 ng/mL) hybrid solution containing probe was added and crossed at 42 °C. After washed by phosphate-buffered saline with Tween (PBST, 0.01 M, pH 7.4) for 3 times, the nucleus were dyed with DAPI solution diluted by PBST (ab104139, 1:100, Abcam, Shanghai, China), then added to the 24-well culture plate and stained for 5 min. Finally, the cells were blocked with antifluorescence quenching agent, and a fluorescence microscope (Olympus, Tokyo, Japan) was adopted to observe and capture the images of cells.

### Dual luciferase reporter gene assay

The target sites of wild type (WT) of miR-34b and TUFT1 mRNA 3′-UTR region and the sequence after site directed mutagenesis from the WT named mutant type (MUT) were synthesized. Restriction endonuclease was used for detachment based on the PmiR-RB-REPORT™ plasmid (RiboBio Co., Ltd., Guangzhou, China). Then the target gene fragments WT and MUT were inserted into pmiR-RB-REPORT™ vector (RiboBio Co., Ltd., Guangzhou, China), respectively. The empty plasmid was simultaneously transferred as the control group while the correct luciferase reporter gene plasmids WT and MUT were utilized to subsequent transfection. The vectors of MUT and WT were co-transferred to 293T cells with mimic-NC or miR-34b mimic together with oe-NC or oe-HNF1A-AS1, respectively. After 48 h transfection, the cells were collected and lysed, and the culture fluid was obtained by centrifugation at 10,000 rpm, 4 °C for 3 min. Relative lights units (RLU) was detected by luciferase detection kit (RG005, Beyotime Biotechnology Co., Ltd, Shanghai, China). Relative fluorescence value was calculated as RLU value determined by renilla luciferase/the RLU value measured by firefly luciferase.

### RNA immunoprecipitation (RIP) assay

RIP kit (Millipore, Bedford, MA, USA) was adopted to detect the combination of lncRNA HNF1A-AS1 and Ago2. With the same volume of phenylmethylsulphonyl fluoride (PMSF) and protease inhibitor, the cells were lysed for 30 min. The supernatant was obtained by centrifugation at 14,000 rpm, 4 °C for 10 min. Part of the cell extract was used as Input and another was precipitated with antibody. Each co-precipitation reaction system was washed with magnetic bead and suspended in 100 μL RIP Wash Buffer, then incubated with 5 μg antibody on the basis of experiment group. The magnetic bead antibody complex was resuspended in 900 μL RIP Wash Buffer and incubated with 100 μL cell extract at 4 °C overnight. The magnetic globin complex was collected on the magnetic pedestal. The samples and Inputs were detached with protease K to extract RNA for PCR detection. The antibodies used in RIP were rabbit anti-Ago2 (ab186733, 1:50, Abcam, Shanghai, China). Rabbit anti-IgG (ab109489, 1:100, Abcam, Shanghai, China) was used as the NC.

### RNA pull-down assay

WT-bio-miR-34b and MUT-bio-miR-34b (GeneCreate Biological Engineering Co., Ltd. Wuhan, China) labeled by 50 nM biotin was used to transfect cells. The cells were collected and washed with PBS (0.01 M, pH 7.4) after 48 h. The cells were incubated in a specific lysis buffer (Ambion, Austin, Texas, USA) for 10 min. M-280 streptavidin beads (S3762, Sigma-Aldrich, St Louis, MO, USA) which pre-coated with RNase-free bovine serum albumin (BSA) and yeast tRNA (TRNBAK-RO, Sigma-Aldrich, St Louis, MO, USA) was incubated with lysate at 4 °C overnight. Cells was washed twice with precooled pyrolysis buffer, 3 times with low salt buffer, and once with high salt buffer. The purification of bound RNA was through Trizol, and the enrichment of lncRNA HNF1A-AS1 was verified by RT-qPCR.

### RT-qPCR

Total RNA was extracted from cells and tissues by Trizol (TaKaRa, Dalian, China) after collection and treatment of the cells in each group. According to the instruction of reverse transcription kit (K1621, Fermentas, Maryland, New York, USA), RNA was reversely transcribed to cDNA. The HNF1A-AS1, miR-34b and TUFT1 primer sequences (Table 1) were designed and synthesized by Shanghai Genechem Co., Ltd (Shanghai, China). Fluorescent quantitative PCR kit (TaKaRa, Dalian, China) was used to detect the mRNA expression of each gene. RT-qPCR (ABI 7500, ABI, Foster City, CA, USA) was used for detection. U6 was used as an internal parameter of miR-34b and glyceraldehyde-3-phosphate dehydrogenase (GAPDH) of HNF1A-AS1 and TUFT1. The relative expression of each target gene was calculated by 2^−ΔΔCt^ method.

**Table 1:** Primer sequence

Gene	Primer sequence (5′-3′)
HNF1A-AS1	F: 5′-TCAAGAAATGGTGGCTAT-3′
	R: 5′-GCTCTGAGACTGGCTGAA-3′
miR-34b	F: 5′-AGTTGAGAAACAAG GGCTCAA-3′
	R: 5′-GTA TCCAGTGCAGG GTCC′
TUFT1	F: 5′-AACGCTTCACGAATTTGCGT’
	R: 5′-GCTTTGCCGAGCCCTATAA-3′
U6	F: 5′-CTCGCTTCGGCAGCACA-3′
	R: 5′-AACGCTTCACGAATTTGCGT-3′
GAPDH	F: 5′-GGGAGCCAAAAGGGTCAT-3′
	R: 5′-GAGTCCTTCCACGATACCAA-3′

*F* forward, *R* reverse, *miR-34b* microRNA-34b, *GAPDH* glyceraldehyde-3-phosphate dehydrogenase

### Western blot assay

RIPA buffer (100 μL) (R0020, Solaibao Technology Co., Ltd., Beijing, China, containing 1 mmoL/L PMSF) was added. The protein concentration was determined by the instruction of bicinchoninic acid kit (AR0146, Boster Biological Technology co. Ltd, Wuhan, Hubei, China). The sample concentration was adjusted to 3 μg/μL. The sample buffer was added into the extracted protein and boiled at 95 °C for 10 min. And then the protein was isolated by 10% polyacrylamide gel electrophoresis. The protein was transferred to polyvinylidene fluoride (PVDF) membrane (p2438, Sigma-Aldrich, St Louis, MO, USA). The membrane was blocked with 5% BSA (10L16, Zhongsheng Likang Technology Co., Ltd., Beijing, China) for 1 h in room temperature. Next, the rabbit anti-CD63 (ab59479, 1:1000), CD9 (ab2215, 1:1000), CD81 (ab79559, 1:1000) (all from Abcam, Cambridge, USA) was added and incubated at 4 °C overnight. After washing by TBST (pH 7.4, 10×, Elabscience Biotechnology Co., Ltd, Wuhan, Hubei, China) 3 times × 5 min, cells were incubated with corresponding goat anti-rabbit secondary antibody (ab6721, 1:2000, Abcam, Cambridge, USA) for 1 h. The membrane was developed through chemiluminescence reagent with GADPH (ab181602, 1:10,000, Abcam, Cambridge, USA) as an internal reference. Gel Doc imager (Bio-rad, California, USA) was used to develop. Eventually, Image J software was used to analyze the gray value of target band.

### Tumor xenografts in nude mice

BALB/c nude mice aged 3–5 weeks old and weighing about 10–12 g were bred in laminar flow cabinet of the barrier system (specific pathogen-free grade). The indoor UV irradiation was carried out regularly. Cage, cushion, drinking water and feed were sterilized under high pressure. The room temperature was controlled at 24–26 °C and the relative humidity was 40–60%. The cultured HeLa cells were taken, and the concentration of cell suspension was adjusted to 1 × 10^6^ cells/mL with PBS and 50 μL of the cell suspension was applied for a subcutaneous injection to the right side of mice. One week later, the mice were randomly assigned into four groups, eight in each group: (1) PBS group; (2) DDP group; (3) DDP + sh-NC group; (4) DDP + sh-HNF1A-AS1 group. After 28 days, the mice were euthanized with pentobarbital sodium for anaesthesia (100 mg/kg, Cat. No. P3761, Sigma-Aldrich, St Louis, MO, USA), the tumor was dissected, the short diameter (a) and long diameter (b) of the tumor were recorded with a ruler. Tumor volume was calculated by π (a^2^b)/6, and tumor weight was evaluated with a balance.

### Statistical analysis

All data were analyzed by SPSS 21.0 software (IBM Corp. Armonk, NY, USA). The measurement data were represented by mean ± standard deviation. Comparisons between two groups were conducted by t-test, while comparisons among multiple groups were assessed by one-way analysis of variance (ANOVA) followed by Tukey’s post hoc test. *P* value < 0.05 was indicative of statistically significant difference.

## Results

### HNF1A-AS1 is elevated in DDP-resistant CC cells

In order to explore the expression of HNF1A-AS1 in DDP-resistant CC cells, we used RT-qPCR to detect the expression of HNF1A-AS1 in human normal cervical epithelial cell line HcerEpic, DDP-sensitive CC cell line (HeLa/S) and DDP-resistant cell line (HeLa/DDP). The results reported that the expression of HNF1A-AS1 elevated in HeLa/DDP cells compared with HcerEpic and HeLa/S cells (*P *< 0.05) (Fig. 1a). This result suggested that HNF1A-AS1 may be involved in drug resistance of CC.

**Fig. 1:** Interfering with HNF1A-AS1 inhibits the drug resistance and proliferation of cervical cancer cells and promotes their apoptosis. **a** Detection of HNF1A-AS1 expression in each cell lines by RT-qPCR. **b** RT-qPCR was used to detect the interference efficiency of HNF1A-AS1 in DDP-sensitive cell line HeLa/S and DDP-resistant cell line HeLa/DDP. **c** Detection of IC_50_ in DDP-sensitive cell line HeLa/S and DDP-resistant cell line HeLa/DDP by MTT assay. **d** EdU assay was adopted to detect cell proliferation of DDP-sensitive cell line HeLa/S and DDP-resistant cell line HeLa/DDP. **e** Colony formation assay detected the ability of cell colony formation of DDP-sensitive cell line HeLa/S and DDP-resistant cell line HeLa/DDP. **f** Flow cytometry was used to detect cell apoptosis of DDP-sensitive cell line HeLa/S and DDP-resistant cell line HeLa/DDP. *P < 0.05 vs. HcerEpic cells. ^#^*P *< 0.05 vs. the sh-NC group. Measurement data were depicted as mean ± standard deviation, comparisons between groups were conducted by non-paired *t* test, and comparisons among multiple groups were assessed by one-way analysis of variance, the experiment was repeated three times

To further validate the role of HNF1A-AS1 in drug resistance of CC, we interfered with HNF1A-AS1 in the HeLa/S and HeLa/DDP cells, and the expression of HNF1A was detected by RT-qPCR. It suggested that the expression of HNF1A-AS1 decreased in the sh-HNF1A-AS1 groups compared with the sh-NC group (*P *< 0.05) (Fig. 1b), and sh-HNF1A-AS1-1 sequence with the lowest expression was selected for subsequent experiments and named as sh-HNF1A-AS1. After that, different groups of cells were processed with DDP, whereas the IC_50_ of HeLa/S and HeLa/DDP was detected by MTT assay. The results suggested that the IC_50_ of the sh-HNF1A-AS1 group was lower than that in the sh-NC group (*P* < 0.05) (Fig. 1c). The EdU assay and colony formation assay were adopted to detect the cell proliferation and colony formation ability of HeLa/S and HeLa/DDP, respectively. The results demonstrated that the cell proliferation and colony formation ability of cells in the sh-HNF1A-AS1 group were lower than that in the sh-NC group (both *P* < 0.05) (Fig. 1d, e). Flow cytometry results showed that the apoptosis of cells in the sh-HNF1A-AS1 group was significantly increased relative to the sh-NC group (*P *< 0.05) (Fig. 1f). These data indicated that interference with HNF1A-AS1 can significantly inhibit the drug resistance, proliferation and promote apoptosis of CC cells.

### Sensitive cells assimilate exosomes from drug-resistant cells

Previous studies have shown that exosomes secreted by breast cancer cells were involved in drug-resistant metastasis [20–22]. Exosomes could be absorbed by breast cancer cells and effectively increased the drug resistance of breast cancer sensitive cell lines [23]. In order to explore the impact of exosomes on cell drug resistance in CC, the exosomes in the culture supernatant of DDP-resistant cell lines were isolated by high-speed centrifugation and observed under a TEM. Presented circular or elliptical membranous vesicle-like vesicles with a diameter of approximately 30–60 nm, it was in accord with the morphological characteristics of the exosomes (Fig. 2a). Dynamic light scattering detection found that the exosome particle diameters ranged from 30 to 120 nm (Fig. 2b). Western blot assay revealed that the white precipitate had the expression of exosome markers CD63, CD9, and CD81 (Fig. 2c), thus confirming that we successfully isolated the exosomes. To verify whether CC sensitive cell lines could absorb drug-resistant exosomes, exosomes and CC sensitive cell lines were co-cultured. The results of laser confocal microscope showed (Fig. 2d) that the green fluorescence of PKH67 was uniformly distributed in the cytoplasm of most of the HeLa/S cells, confirming that the HeLa/S cells can effectively uptake the exosomes of the drug-resistant cells.

**Fig. 2:** Drug-resistant exosomes can be absorbed by sensitive cells. **a** The morphological characteristics of exosomes by a transmission electron microscope. **b** The diameter of exosomes detected by dynamic light scattering. **c** Exosomes surface marker protein CD63, CD9 and CD81 detected by western blot analysis. **d** Fluorescence labeled and uptake exosomes through a laser confocal microscopy (×400). The experiment was repeated three times

### DDP-exo affects cell proliferation, apoptosis and drug resistance by promoting HNF1A-AS1 expression

In order to further study the involvement of exosomes in CC drug-resistant metastasis, we extracted the exosomes of different cells and HeLa/S cells, and then treated with DDP for 48 h, then MTT assay was utilized to detect the IC_50_ of HeLa/S cells. The results showed (Fig. 3a) that the IC_50_ in the HeLa/S + DDP-exo group was significantly increased (*P *< 0.05), while the HeLa/S + S-exo group had no significant change relative to the HeLa/S group (*P *> 0.05). Then, the proliferation of HeLa/S and the apoptosis of cells in different groups was detected by EdU assay and flow cytometry, respectively. The results revealed that (Fig. 3b, c), the cell proliferation in the HeLa/S + DDP-exo group increased significantly, and there was also a significant decrease in cell apoptosis (both *P *< 0.05), while the HeLa/S + S-exo group relative to the HeLa/S group had no significant difference (*P *> 0.05). This result indicated that exosomes from drug-resistant cells could transmit drug resistance to drug-sensitive cells. Exosomes of drug-sensitive cells did not affect their own cells. The expression of HNF1A-AS1 in each group was detected by RT-qPCR. The results revealed that (Fig. 3d), in contrast with the HeLa/S group, the expression of HNF1A-AS1 was increased in the HeLa/S + DDP-exo group (*P *< 0.05). This result indicated that DDP-exo promoted HNF1A-AS1 expression to affect cell proliferation, apoptosis and drug resistance of CC cells.

**Fig. 3:** DDP-exo promotes HNF1A-AS1 expression to affect cervical cancer cell proliferation, apoptosis and drug resistance. **a** MTT assay was used to detect IC_50_ of DDP-treated cells in each group. **b** EdU assay was used to detect the proliferation of DDP-treated cells. **c** Flow cytometry was used to detect apoptosis of DDP-treated cells. **d** RT-qPCR was used to detect the expression of HNF1A-AS1 in each group of cells. *P < 0.05 vs. the HeLa/S group. Measurement data were depicted as mean ± standard deviation, comparisons among multiple groups were assessed by one-way analysis of variance, the experiment was repeated three times

### HNF1A-AS1 acts as a ceRNA of miR-34b to promote TUFT1 expression

To investigate the mechanism of HNF1A-AS1, FISH assay was applied for detecting the subcellular localization of HNF1A-AS1, and the results revealed that HNF1A-AS1 was concentrated in the cytoplasm (Fig. 4a), suggesting that HNF1A-AS1 may function in the cytoplasm. Through the RNA22 website (https://cm.jefferson.edu/rna22/Precomputed/), it revealed that HNF1A-AS1 could bind to miR-34b (Fig. 4b), and further verified by dual luciferase reporter gene assay: in contrast to the oe-NC group, the luciferase activity of WT-miR-34b/oe-HNF1A-AS1 was decreased in the oe-HNF1A-AS1 group (*P* < 0.05); and the luciferase activity of MUT-miR-34b/oe-HNF1A-AS1 showed no significant difference (*P* > 0.05), indicating that miR-34b may specifically bind to HNF1A-AS1 (Fig. 4c). RIP assay was adopted to detect the relationship between HNF1A-AS1 and Ago2, and it demonstrated that the specific adsorption level of HNF1A-AS1 to Ago2 was higher than that in the IgG group (*P* < 0.05) (Fig. 4d). The RNA pull-down assay was used to verify whether HNF1A-AS1 could be used as a ceRNA to adsorb miR-34b. The results revealed that the enrichment level of HNF1A-AS1 was increased in the Bio-miR-34b-WT group (*P* < 0.05), but there was no obvious difference in the enrichment level of HNF1A-AS1 in the Bio-miR-34b-MUT group (*P* > 0.05) in contrast to the Bio-probe NC group (Fig. 4e). These results indicated that lncRNA HNF1A-AS1 could adsorb miR-34b as a ceRNA, thereby affecting the expression of miR-34b.

**Fig. 4:** HNF1A-AS1 acts as a ceRNA of miR-34b to promote the expression of TUFT1. **a** FISH assay verify HNF1A-AS1 subcellular localization. **b** RNA22 site predicts binding sites of HNF1A-AS1 and miR-34b. **c** Dual luciferase reporter gene assay was performed to verify the binding of HNF1A-AS1 to miR-34b. **d** The binding of HNF1A-AS1 to Ago2 detected by RIP assay. **e** RNA pull-down assay detected the enrichment of HNF1A-AS1 by miR-34b. **f** RT-qPCR detected the expression of miR-34b in DDP-sensitive cell line HeLa/S and DDP-resistant cell line HeLa/DDP. **g** Prediction of targeting relationship between miR-34b and TUFT1 in RNA22 website. **h** The targeting relationship between miR-34b and TUFT1 using luciferase activity assay. **i** Detection of TUFT1 expression in DDP-sensitive cell line HeLa/S and DDP-resistant cell line HeLa/DDP using RT-qPCR. *P < 0.05. Measurement data were depicted as mean ± standard deviation, and comparisons between groups were conducted by non-paired *t* test, and comparisons among multiple groups were assessed by one-way analysis of variance, the experiment was repeated three times

Therefore, we further used RT-qPCR to verify the expression of miR-34b in DDP sensitive cells and DDP resistant CC cells. The results demonstrated that miR-34b was poorly expressed in HeLa/DDP cells (Fig. 4f). The target gene of miR-34b was predicted in RNA22 website, it was found that there existed a binding site between miR-34b and TUFT1 (Fig. 4g). Also, we found in dual luciferase reporter gene assay that (Fig. 4h) TUFT1 was the target gene of miR-34b (*P *< 0.05). RT-qPCR tested the expression of TUFT1 in HeLa/S and HeLa/DDP cells. The results demonstrated that TUFT1 was up-regulated in HeLa/DDP cells (*P* < 0.05) (Fig. 4i). It was speculated that HNF1A-AS1 may act as ceRNA to adsorb miR-34b, and then the expression of miR-34b was inhibited, finally, the expression of TUFT1 was up-regulated.

### Exosomes shuttled HNF1A-AS1 down-regulates miR-34b and up-regulates TUFT1 expression to promote the proliferation and drug resistance as well as inhibit apoptosis of CC cells

The aforementioned studies indicated that the exosomes secreted by HeLa/DDP cells can transmit drug resistance. To further investigate whether drug-resistant exosomes could promote drug resistance through modulating expression of HNF1A-AS1, we established a co-culture model to study the effect of exosomal HNF1A-AS1 on DDP sensitive cells. The DDP resistant cells transfected with overexpression HNF1A-AS1 plasmid marked by Cy3 were co-cultured with DDP sensitive cells for 24 h, and then the effects on IC_50_, proliferation and apoptosis of DDP sensitive cells were detected. The results displayed (Fig. 5a–c) that in relation to the NC-exo group, the IC_50_ and proliferation of the HNF1A-AS1-exo group had a obviously increase and a obviously decrease in the apoptotic rate (all *P* < 0.05). In order to know that expression of miR-34b and TUFT1 in the cells after the expression of HNF1A-AS1-exo, RT-qPCR was used and the results were shown (Fig. 5d) that after overexpression of HNF1A-AS1-exo by donor cells, miR-34b was down-regulated and TUFT1 was up-regulated (both *P* < 0.05). All these data suggested that exosomes shuffled HNF1A-AS1 promoted proliferation and drug-resistance and suppressed the apoptosis of CC cells through down-regulation of miR-34b and up-regulation of TUFT1.

**Fig. 5:** Exosomes shuttled HNF1A-AS1 down-regulates miR-34b and upregulates TUFT1 expression to promote the proliferation, drug resistance, and inhibit apoptosis of cervical cancer cells. **a** MTT assay was used to detect IC_50_ of DDP-treated cells in each group; **b** proliferation of DDP-treated cells using EdU assay. **c** Flow cytometry was used to detect apoptosis of DDP-treated cells. **d** RT-qPCR was used to detect the expression of miR-34b and TUFTI after overexpression of HNF1A-AS1-exo. *P < 0.05 vs. the NC-exo group. Measurement data were depicted as mean ± standard deviation, comparisons between groups were conducted by non-paired *t* test. The experiment was repeated three times

### Inhibition of exosomal HNF1A-AS1 in HeLa/DDP combined with DDP inhibited tumor formation in nude mice

In order to elucidate the effect of exosomal HNF1A-AS1 in HeLa/DDP cells combined with DDP on tumor formation in nude mice, we first constructed a subcutaneous tumor formation model of nude mice with HeLa cells, which were treated differently after tumor formation. Tumor growth curves and tumor weight measurements showed that the volume and weight of tumors in mice were significantly reduced after DDP treatment (*P* < 0.05). Compared with the DDP + sh-NC group, the weight and volume of tumors were significantly reduced in the DDP + sh-HNF1A-AS1 group (both *P* < 0.05) (Fig. 6a–c). This result suggested that tumor formation in nude mice can be suppressed by inhibiting exosomal HNF1A-AS1 in combination with DDP.

**Fig. 6:** Inhibited exosomal HNF1A-AS1 in DDP-resistant cells HeLa/DPP combined with DDP inhibited tumor formation in nude mice. **a** The subcutaneous tumor growth curve of each group of nude mice (n = 8). **b** The tumor weight comparison histogram of each group in nude mice (n = 8). **c** Tumor of nude mice in tumor xenografts experiment. Measurement data were depicted as mean ± standard deviation, and comparisons between two groups were assessed by non-paired *t* test

## Discussion

Cervical cancer is one of the main causes of cancer death in women [22]. Moreover, the expression of miR-34b was poorly expressed in CC samples, and cell migration could be inhibited by miR-34b whereas cell apoptosis could be induced by regulating TGF-1 [16]. It had also been verified that TUFT1 is expressed in some cancers and participates in the proliferation and survival of cancers cells [18]. As the related mechanisms of HNF1A-AS1 in CC remains to be excavated, our study was to inquiry the effect of exosomal lncRNA HNF1A-AS1 in CC and it inner mechanisms.

In this study, it was found that an overexpression of HNF1A-AS1 in DDP-resistant CC cells and depletion of HNF1A-AS1 markedly inhibited the drug resistance, proliferation and promoted apoptosis of CC cells. In a current study, an analysis to the next generation sequencing of human esophageal tissue demonstrated that HNF1A-AS1 was significantly highly expressed in oesophageal adenocarcinoma tissue compared with the normal esophagus [24]. Likewise, another study has revealed an up-regulation of HNF1A-AS1 in non-small cell lung cancer (NSCLC) [25]. A study has shown an overexpression of HNF1A-AS1 in gastric cancer tissues, while the low expression of HNF1A-AS1 could suppress the proliferation of gastric cancer cells [7]. Furthermore, similar to our study, the down-regulation of HNF1A-AS1 significantly inhibited the proliferation, invasion, migration and colony formation of colorectal cancer cells, and inhibited the entry of S phase in vitro [26]. Additionally, the finding from our investigation showed that DDP-exo affects cell proliferation, apoptosis and drug resistance by promoting HNF1A-AS1 expression. There are some studies concentrated on the relationship between exosomes and lncRNAs. For example, a research has provided a proof that the exosomes derived from endothelial progenitor cells can promote the regeneration and differentiation of osteoclast precursors through lncRNA MALAT1, thereby promoting bone repair [27]. It has been showed that expression of the lncRNA GAS5 in secreted exosomes is elevated and exosomes can dynamically monitor the level of GAS5 [28]. Another article has suggested that lncRNA ATB may exert an enormous function on the regulation of the microenvironment of glioma by exosomes [29].

Moreover, we demonstrated that HNF1A-AS1 acted as a ceRNA of miR-34b to promote TUFT1 expression. A study has indicated that HNF1A-AS1 promotes autophagy and carcinogenesis by sponging miR-30b, whereas HNF1A-AS1 and its corresponding ceRNAs have the same miRNA response elements as miR-30b [30]. Another study has suggested that the HNF1A-AS1 may as a ceRNA in the NSCLC cells to sponge miR-17-5p. In addition, the HNF1A-AS1/miR-17-5p axis is considered as a promising target for the treatment of NSCLC [31]. Interestingly, a previous research has demonstrated that hypoxia/HIF-1α signaling increases the expression of TUFT1 through downregulating miR-671-5p [17].

Our data also suggested that exosomes shuttled HNF1A-AS1 downregulates miR-34b and upregulates TUFT1 expression to promote the proliferation and drug resistance as well as inhibit apoptosis of CC cells. A study has presented that miR-34b expression was dramatically reduced in CC relative to that in the adjacent normal tissues while restored miR-34b attenuated cell proliferation and facilitated the apoptosis of CC cell lines [16]. Another study revealed that the expression of TUFT1 was heightened in breast cancer samples while down-regulation of TUFT1 decreased proliferation and increased apoptosis of breast cancer cells [18]. Furthermore, an experiment in vivo suggested that inhibition of exosomal HNF1A-AS1 in HeLa/DDP combined with DDP inhibited tumor formation in nude mice. The results of in vivo experiment was in accordance with the results of in vitro experiments.

## Conclusion

Overall, our results suggest that exosomes carrying HNF1A-AS1 as a ceRNA of miR-34b to promote the expression of TUFT1 and the drug resistance of CC cells. Our work identified a new clue for further investigating the pathogenesis of CC. The results of this paper can be further verified by expanding the sample size in the future.

## Data Availability

Not applicable.

## Abbreviations

lncRNAs: long-term non-coding RNAs
CC: cervical cancer
HPV: human papillomavirus
RT: radiotherapy
RHND: radical hysterectomy with pelvic lymph node dissection
HNF1A-AS1: HNF1A antisense RNA 1
miRNA: microRNA
ceRNA: competing endogenous RNA
TUFT1: tuftelin1
FBS: fetal bovine serum
RIPA: radioimmunoprecipitation assay
BCA: bicinchoninic acid
TEM: transmission electron microscope
RT-qPCR: reverse transcription quantitative polymerase chain reaction
EdU: 5-ethynyl-2′-deoxyuridine
EDTA: ethylene diamine tetraacetic acid
FISH: fluorescence in situ hybridization
PBST: phosphate-buffered saline with Tween
WT: wild type
3′-UTR: 3′-untranslated region
MUT: mutant type
NC: negative control
RLU: relative lights units
RIP: RNA immunoprecipitation
PMSF: phenylmethylsulphonyl fluoride
BSA: bovine serum albumin
GAPDH: glyceraldehyde-3-phosphate dehydrogenase
PVDF: polyvinylidene fluoride
ANOVA: one-way analysis of variance
NSCLC: non-small cell lung cancer
